The article "Long Noncoding RNA FOXD2-AS1 Promotes the Malignancy of Cervical Cancer by Sponging MicroRNA-760 and Upregulating Hepatoma-Derived Growth Factor" was retracted in 2023. Reasons: duplicated images; signs of a paper mill; original data or images not available; unreliable results or conclusions.

# Long Noncoding RNA *FOXD2-AS1* Promotes the Malignancy of Cervical Cancer by Sponging MicroRNA-760 and Upregulating Hepatoma-Derived Growth Factor

**DOI:** 10.3389/fphar.2019.01700

**Published:** 2020-01-31

**Authors:** Xiaoqing Dou, Qun Zhou, Mingxiao Wen, Jiangyan Xu, Yingping Zhu, Shuzhen Zhang, Xianli Xu

**Affiliations:** ^1^ Department of Gynecology, The First Affiliated Hospital of Zhejiang Chinese Medical University, Zhejiang Provincial Hospital of Traditional Chinese Medicine, Hangzhou, China; ^2^ Department of Clinical Laboratory, The First Affiliated Hospital of Zhejiang Chinese Medical University, Zhejiang Provincial Hospital of Traditional Chinese Medicine, Hangzhou, China

**Keywords:** cervical cancer, microRNA-760, hepatoma-derived growth factor, FOXD2 adjacent opposite strand RNA 1, *FOXD2-AS1*

## Abstract

Although the functions of long noncoding RNA (lncRNA) called FOXD2 adjacent opposite strand RNA 1 (*FOXD2-AS1*) have been well studied in multiple human cancer types, its expression status and detailed roles in cervical cancer remain unknown and merit investigation. This study was aimed at assessing *FOXD2-AS1* expression in cervical cancer and at determining its effects on the aggressive behavior of cervical cancer *in vitro* and *in vivo*. Expression of *FOXD2-AS1* in cervical cancer tissues and cell lines was determined *via* reverse-transcription quantitative PCR. The effects of *FOXD2-AS1* on cervical cancer cells were examined by a 3-(4,5-dimethyl-2-thiazolyl)-2,5-diphenyl-2-H-tetrazolium bromide (MTT) assay, flow-cytometric analysis, migration and invasion assays, and an *in vivo* tumorigenicity assay. *FOXD2-AS1* was found to be significantly upregulated in cervical cancer tissues and cell lines. High *FOXD2-AS1* expression was notably linked with the Federation of Gynecology and Obstetrics (FIGO) stage, lymph node metastasis, and depth of cervical invasion in patients with cervical cancer. Kaplan–Meier survival analysis revealed significantly shorter overall survival of patients when the tumor expression of *FOXD2-AS1* was higher in comparison with those in patients with lower *FOXD2-AS1* expression. *In vitro* functional assays revealed that downregulation of *FOXD2-AS1* led to suppression of proliferation, migration, and invasiveness as well as to the induction of apoptosis of cervical cancer cells. In addition, *FOXD2-AS1* silencing hindered tumor growth *in vivo*. Mechanism investigation revealed that *FOXD2-AS1* functioned as a molecular sponge of microRNA-760 (miR-760). Furthermore, hepatoma-derived growth factor (*HDGF*) was validated as a direct target gene of miR-760 in cervical cancer cells. Moreover, an miR-760 knockdown reversed the effects of *FOXD2-AS1* silencing on cervical cancer cells. *FOXD2-AS1* possesses significant oncogenic activity in cervical cancer progression; this activity is mediated by sponging of miR-760 with consequent upregulation of HDGF. The *FOXD2-AS1*–miR-760–HDGF axis might harbor promising targets for novel treatment strategies of cervical cancer.

The article "Long Noncoding RNA FOXD2-AS1 Promotes the Malignancy of Cervical Cancer by Sponging MicroRNA-760 and Upregulating Hepatoma-Derived Growth Factor" was retracted in 2023. Reasons: duplicated images; signs of a paper mill; original data or images not available; unreliable results or conclusions.

## Introduction

Cervical cancer is the second most prevalent cancer among women and the fourth leading cause of gynecological-cancer–associated deaths globally (Torre et al., 2015). Approximately 530,000 new cases are expected every year, and 275,000 deaths are caused by cervical cancer worldwide annually (Arbyn et al., 2011). Over 75% of these new cases and deaths occur in developing countries, including China (Barra et al., 2017). Multiple factors, including early sexual intercourse, an increased number of sexual partners, and persistent human papillomavirus infection, have been implicated in the pathogenesis of cervical cancer (Bosch and de Sanjose, 2003; Yu et al., 2013); however, the detailed mechanisms behind the progression of cervical cancer remain largely unclear and need further elucidation. Despite considerable progress in the diagnostic and therapeutic modalities in recent years, the clinical outcomes of patients with cervical cancer unfortunately remain unsatisfactory (Ghebre et al., 2017). The 5-year survival rate of patients with cervical cancer diagnosed at advanced stages is less than 40%, which may be attributable to metastasis and tumor recurrence (Smith et al., 2013; Kogo et al., 2015). Therefore, elucidation of the mechanisms underlying cervical carcinogenesis and cancer progression is crucial and may facilitate identification of novel therapeutic targets to improve the prognosis of patients with cervical cancer.

Long noncoding RNAs (lncRNAs) are a group of RNA molecules with a length of >200 nucleotides that do not encode proteins (Batista and Chang, 2013). LncRNAs are widely expressed in nearly all organs and are implicated in a variety of biological and pathological processes (Ponting et al., 2009). They can function as molecular sponges, scaffolds, and guides for interactions with proteins, mRNAs, or microRNAs (miRNAs), thereby regulating the expression of target genes (Anastasiadou et al., 2018). Accumulated evidence indicates that many lncRNAs are aberrantly expressed in cervical cancer (Chen et al., 2019; Zhang Y. et al., 2019; Zhang X. et al., 2019). Alterations in the expression of lncRNAs are involved in cervical carcinogenesis and cancer progression by playing tumor-suppressive or oncogenic roles (Aalijahan and Ghorbian, 2019). Hence, an in-depth understanding of novel lncRNAs associated with the aggressive behaviors of cervical cancer may contribute to the development of attractive targets for anticancer therapy.

The article "Long Noncoding RNA FOXD2-AS1 Promotes the Malignancy of Cervical Cancer by Sponging MicroRNA-760 and Upregulating Hepatoma-Derived Growth Factor" was retracted in 2023. Reasons: duplicated images; signs of a paper mill; original data or images not available; unreliable results or conclusions.

MiRNAs are a subset of endogenous, single-strand, noncoding small RNAs ranging in size from 17 to 21 nucleotides (Kloosterman and Plasterk, 2006). MiRNAs regulate gene expression by interacting with the complementary sequences in the 3′ untranslated region (3′-UTR) of a target mRNA and by triggering translation suppression and/or mRNA degradation (Bartel, 2009). One mRNA can be directly targeted by numerous miRNAs, and one miRNA is likely to target numerous mRNAs (Zang et al., 2016). MiRNAs are aberrantly expressed in nearly all human cancer types, including cervical cancer (Mandujano-Tinoco et al., 2018; Srivastava et al., 2017; Sharma and Baruah, 2018). MiRNAs may function either as oncomiRs or tumor suppressor miRNAs depending on their target genes (Xia et al., 2016). In particular, a wide range of miRNAs are dysregulated in cervical cancer and are involved in the modulation of various pathological and physiological phenomena, including cell proliferation, the cell cycle, apoptosis, metastasis, angiogenesis, and chemoresistance (Feng et al., 2017; Li et al., 2017; Laengsri et al., 2018). Therefore, miRNAs may be promising therapeutic targets for the management of cervical cancer.

*FOXD2-AS1* is dysregulated in multiple types of human cancer, and its dysregulation is involved in the modulation of various tumor-associated biological processes (Rong et al., 2017; Bao et al., 2018; Chang et al., 2018; Su et al., 2018; Zhang et al., 2018; Zhao et al., 2018; Zhu et al., 2018; Jiang et al., 2019; Liu et al., 2019; Ni et al., 2019; Ren et al., 2019; Xu et al., 2019). To the best of our knowledge, however, the expression status and detailed roles of *FOXD2-AS1* in cervical cancer are still unknown. Therefore, the objectives of this study were to evaluate *FOXD2-AS1* expression in cervical cancer, investigate the effects of *FOXD2-AS1* on cervical cancer cells, and elucidate the potential mechanism underlying these effects. Our study identified a novel pathway, *FOXD2-AS1*–miR-760–HDGF, involved in cervical cancer progression.

## Materials and Methods

### Clinical Tissue Samples

In total, 63 pairs of cervical cancer tissue samples and adjacent noncancerous tissues were collected from patients with cervical cancer who underwent surgical resection in The First Affiliated Hospital of Zhejiang Chinese Medical University. None of the patients underwent chemotherapy, radiotherapy, or other anticancer therapy prior to the surgical procedure. Tissue specimens were quickly snap-frozen in liquid nitrogen after the surgical resection and then transferred to a −80°C freezer for storage until RNA extraction. The study protocol was approved by the Ethics Committee of The First Affiliated Hospital of Zhejiang Chinese Medical University. Written informed consent was provided by all participants before the collection of tissue samples.

The article "Long Noncoding RNA FOXD2-AS1 Promotes the Malignancy of Cervical Cancer by Sponging MicroRNA-760 and Upregulating Hepatoma-Derived Growth Factor" was retracted in 2023. Reasons: duplicated images; signs of a paper mill; original data or images not available; unreliable results or conclusions.

### Cell Lines and Culture Conditions

A normal human cervix epithelial cell line (Ect1/E6E7) was acquired from the American Type Culture Collection (Manassas, VA, USA). Four human cervical cancer cell lines (HeLa, C-33A, SiHa, and CaSki) were ordered from the Shanghai Institute of Biochemistry and Cell Biology (Shanghai, China). Dulbecco’s modified Eagle’s medium (DMEM) supplemented with 10% (v/v) of heat-inactivated fetal bovine serum (FBS) and 1% (v/v) of a penicillin/streptomycin solution (all from Gibco; Thermo Fisher Scientific, Inc., Waltham, MA, USA) was used to culture all the above cell lines. All cells were grown at 37°C in a humidified incubator supplied with 5% CO_2_.

### A Gene Knockdown and Overexpression

The mimic, negative control mimic (miR-NC), inhibitor, and NC inhibitor for miR-760 were obtained from GenePharma Co., Ltd. (Shanghai, China). For a *FOXD2-AS1* knockdown, small interfering RNA (siRNA) was used (si-FOXD2-AS1); this oligo and negative control siRNA (NC siRNA) were chemically synthesized by RiboBio Co., Ltd. (Guangzhou, China). For HDGF upregulation, HDGF overexpression plasmid pcDNA3.1-HDGF (pc-HDGF) and the empty pcDNA3.1 vector were purchased from the Chinese Academy of Sciences (Changchun, China). Approximately 12 h before transfection, cells were seeded in 6-well plates. The above-mentioned oligos were transfected into the cells by means of Lipofectamine 2000 (Invitrogen, Carlsbad, CA, USA) in accordance with the manufacturer’s protocol.

### RNA Extraction and Reverse-Transcription Quantitative PCR (RT-qPCR)

The TRIzol reagent (Invitrogen, Carlsbad, CA, USA) was utilized to isolate total RNA from tissue specimens or cells in line with the manufacturer’s protocol. The concentration of total RNA was measured on a NanoDrop Spectrophotometer (NanoDrop Technologies; Thermo Fisher Scientific, Inc.). Total RNA was converted into cDNA using the miScript Reverse Transcription Kit (Qiagen GmbH, Hilden, Germany). The synthesized cDNA was used for the quantification of miR-760 expression with the miScript SYBR Green PCR Kit (Qiagen GmbH). Internal control for miR-760 was U6 small nuclear RNA. To analyze *FOXD2-AS1* and HDGF mRNA expression, reverse transcription was conducted with the PrimeScript RT Reagent Kit (Takara Biotechnology Co., Ltd., Dalian, China). Next, qPCR was carried out with SYBR Premix Ex Taq^™^ (Takara Biotechnology Co., Ltd.). *GAPDH* served as an internal reference for *FOXD2-AS1* and HDGF. Relative gene expression was calculated by the 2^−ΔΔCt^ method (Livak and Schmittgen, 2001).

The article "Long Noncoding RNA FOXD2-AS1 Promotes the Malignancy of Cervical Cancer by Sponging MicroRNA-760 and Upregulating Hepatoma-Derived Growth Factor" was retracted in 2023. Reasons: duplicated images; signs of a paper mill; original data or images not available; unreliable results or conclusions.

### A 3-(4,5-Dimethyl-2-Thiazolyl)-2,5-Diphenyl-2-H-Tetrazolium Bromide (MTT) Assay

Transfected cells were collected after 24 h of incubation and seeded separately in 96-well plates at a density of 3,000 cells/well. The cells were then incubated at 37°C and 5% CO_2_. The MTT assay was performed at four time points as follows: 0, 24, 48, and 72 h after cell seeding. In particular, 20 µl of the MTT reagent (5 mg/ml; Sigma-Aldrich; Merck KGaA, Darmstadt, Germany) was added into each well, and the cells were incubated at 37°C and 5% CO_2_ for another 4 h. After that, the culture medium was removed followed by the addition of 200 µl of dimethyl sulfoxide (Sigma-Aldrich; Merck KGaA, Darmstadt, Germany) to dissolve the violet formazan crystals. Finally, a microplate reader (Bio-Rad Laboratories, Hercules, CA, USA) was employed to measure optical density at 490 nm wavelength.

### Flow-Cytometric Analysis

Transfected cells were collected after 48 h of incubation. The proportion of apoptotic cells was determined with the Annexin V-Fluorescein Isothiocyanate (FITC) Apoptosis Detection Kit (BioLegend, Inc., San Diego, CA, USA). Briefly, ice-cold phosphate-buffered saline (PBS; Gibco; Thermo Fisher Scientific, Inc.) was utilized to wash the transfected cells. The cells were then resuspended in 100 µl of 1× binding buffer which was supplemented with 5 µl of Annexin V-FITC and 5 µl of a propidium iodide (PI) solution. Flow cytometry (FACScan™, BD Biosciences, Franklin Lakes, NJ, USA) was conducted to evaluate the apoptosis rate by detecting the proportion of Annexin V-FITC-positive-PI-negative cells.

### Migration and Invasion Assays

After 48 h of transfection, the invasive ability of cervical cancer cells was examined by means of 24-well Transwell chambers (24-well insert; pore size: 8 µm; Corning Inc., Corning, NY, USA) precoated with Matrigel (BD Biosciences). Briefly, transfected cells were harvested and resuspended in the FBS-free culture medium. In total, 5 × 10^4^ cells were seeded in the upper compartment of each insert, while the lower compartment was filled with 500 µl of DMEM containing 20% of FBS. After 24 h incubation, noninvading cells were gently removed by swabbing the top layer of Matrigel with a cotton swab. The invading cells adhering to the undersurface of the insert were fixed with 100% methanol followed by staining with 0.5% crystal violet and washing with PBS. The invasive ability was assessed by counting the invading cells in five randomly chosen visual fields per insert under a light microscope (200× magnification; Olympus Corporation, Tokyo, Japan). The migration assay was carried out according to the experimental procedures similar to those of the invasion assay, except that the chambers were not coated with Matrigel.

The article "Long Noncoding RNA FOXD2-AS1 Promotes the Malignancy of Cervical Cancer by Sponging MicroRNA-760 and Upregulating Hepatoma-Derived Growth Factor" was retracted in 2023. Reasons: duplicated images; signs of a paper mill; original data or images not available; unreliable results or conclusions.

### An *In Vivo* Tumorigenicity Assay

Four-week-old female BALB/c nude mice were ordered from Shanghai SLAC Laboratory Animal Co., Ltd., (Shanghai, China). HeLa cells transfected with si-FOXD2-AS1 or si-NC were subcutaneously injected into the flank of nude mice. The width and length of tumor xenografts were measured every 2 days. Four weeks after injection, all the nude mice were euthanized, after which the tumor xenografts were excised and weighed. The volumes of tumor xenografts were calculated using the following formula: (length × width^2^)/2. The procedures of the animal experiments were approved by the Institutional Animal Care and Use Committee of The First Affiliated Hospital of Zhejiang Chinese Medical University. All the animal experiments were conducted in accordance with the Animal Protection Law of the People’s Republic of China-2009.

### Target Prediction and a Luciferase Reporter Assay

starBase 3.0 (http://starbase.sysu.edu.cn/) was utilized to search for the miRNAs that could be sponged by *FOXD2-AS1*. Three bioinformatics tools, TargetScan7.1 (http://www.targetscan.org/), miRDB (http://mirdb.org/), and starBase 3.0, were employed to predict the potential targets of miR-760.

For a luciferase reporter assay, the 3′-UTR fragments of *HDGF* containing the wild-type (WT) miR-760–binding sequences and a corresponding mutant (MUT) 3′-UTR fragment were designed and chemically synthesized by Shanghai GenePharma and subcloned into pMIR-REPOR (Promega Corp., Madison, WI, USA). The generated luciferase plasmids were designated as HDGF-WT and HDGF-MUT, respectively. The luciferase plasmids, FOXD2-AS1-WT and FOXD2-AS1-MUT, were chemically synthesized in the same way. Cotransfection with the luciferase plasmid and either the miR-760 mimic or miR-NC into cells was performed using the Lipofectamine 2000 reagent following the manufacturer’s instructions. Luciferase activities were determined at 48 h after cell transfection by means of a Dual-Luciferase Reporter Assay System (Promega Corp.). The relative luciferase activity was normalized to *Renilla* luciferase activity.

### RNA Immunoprecipitation (RIP) Assay

The Magna RIP RNA-Binding Protein Immunoprecipitation Kit (Millipore, Bedford, MA, USA) was used for the RIP assay. Briefly, cells were harvested and lysed with RIP lysis buffer. Next, incubation of 100 μl of the cell extract and RIP buffer containing magnetic beads conjugated to an anti-Argonaute 2 (AGO2) antibody (Millipore) or IgG antibody (Millipore) was performed. To remove the protein, proteinase K was applied to treat the samples, after which the immunoprecipitated RNA was extracted and subjected to RT-qPCR for the measurement of *FOXD2-AS1* and miR-760 expression.

The article "Long Noncoding RNA FOXD2-AS1 Promotes the Malignancy of Cervical Cancer by Sponging MicroRNA-760 and Upregulating Hepatoma-Derived Growth Factor" was retracted in 2023. Reasons: duplicated images; signs of a paper mill; original data or images not available; unreliable results or conclusions.

### Protein Extraction and Western Blot Analysis

Total protein was extracted from transfected cells after 72 h of incubation using ice-cold radioimmunoprecipitation assay buffer (Invitrogen; Thermo Fisher Scientific, Inc.). The concentration of total protein was measured with the BCA Protein Assay Kit (Shanghai Qcbio Science and Technologies Co., Ltd., Shanghai, China). Equal amounts of protein samples were loaded onto each lane for SDS-PAGE, followed by transfer onto polyvinylidene difluoride membranes (Beyotime Institute of Biotechnology, Haimen, China). After blockage at room temperature with 5% dried skimmed milk diluted in Tris-buffered saline containing 0.1% of Tween 20 for 1 h, the membranes were incubated with a rabbit anti-human HDGF monoclonal antibody (1:1000 dilution; cat. # ab128921; Abcam, Cambridge, UK) and a rabbit anti-human GAPDH monoclonal antibody (1:1000 dilution; ab181603; Abcam) overnight at 4°C and next probed with a goat anti-rabbit IgG antibody (horseradish peroxidase conjugate; 1:5000 dilution; ab205718; Abcam) (secondary antibody) at room temperature for 1 h. The protein signals were visualized with the Enhanced Chemiluminescence Kit (Pierce; Thermo Fisher Scientific, Inc.) according to the manufacturer’s protocol.

### Statistical Analysis

Data were presented as the mean ± standard deviation. The χ^2^ test was performed to investigate the correlation between *FOXD2-AS1* expression and clinical parameters among the patients with cervical cancer. Differences between two groups were analyzed by Student’s *t* test. One-way analysis of variance, followed by the Student–Newman–Keuls *post hoc* test, was conducted to evaluate the differences between more than two groups. Expression of *FOXD2-AS1*, miR-760, and *HDGF* tested from cervical cancer tissues and adjacent noncancerous tissue samples was analyzed with paired t-tests. The expression correlations between miR-760 and *HDGF* mRNA levels or between *FOXD2-AS1* and miR-760, were assessed by Spearman’s correlation analysis. Kaplan–Meier survival analysis was carried out to assess patients’ survival. Data with P < 0.05 were assumed to indicate a statistically significant difference.

## Results

### Upregulation of *FOXD2-AS1* Is Linked to Poor Survival Among Patients With Cervical Cancer

To reveal the expression pattern of *FOXD2-AS1* in cervical cancer, we detected its expression in 63 pairs of cervical cancer tissue samples and adjacent noncancerous tissue samples by RT-qPCR. The results showed that *FOXD2-AS1* was significantly upregulated in cervical cancer tissues when compared with noncancerous tissues (**Figure 1A**, P < 0.05). To evaluate the clinical significance of *FOXD2-AS1* in cervical cancer, we subdivided all patients with cervical cancer into low- and high-*FOXD2-AS1* groups based on a median level of *FOXD2-AS1* expression and then investigated the association between *FOXD2-AS1* and the clinical parameters of patients with cervical cancer. Statistical analysis revealed that high *FOXD2-AS1* levels strongly correlated with the International Federation of Gynecology and Obstetrics (FIGO) stage (P = 0.045), lymph node metastasis (P = 0.023), and depth of cervical invasion (P = 0.036) among the patients with cervical cancer (**Table 1**). Notably, Kaplan–Meier survival analysis revealed significantly shorter overall survival when the expression of *FOXD2-AS1* was higher than when this expression was lower (**Figure 1B**, P = 0.019). To further validate the correlation of *FOXD2-AS1* with cervical cancer, *FOXD2-AS1* expression was measured in four cervical cancer cell lines (HeLa, C-33A, SiHa, and CaSki) and a normal human cervix epithelial cell line (Ect1/E6E7) by the same method. The expression level of *FOXD2-AS1* was considerably higher in all four cervical cancer cell lines than in Ect1/E6E7 cells (**Figure 1C**, P < 0.05). These findings suggested that *FOXD2-AS1* may be closely related to the aggressiveness of cervical cancer.

The article "Long Noncoding RNA FOXD2-AS1 Promotes the Malignancy of Cervical Cancer by Sponging MicroRNA-760 and Upregulating Hepatoma-Derived Growth Factor" was retracted in 2023. Reasons: duplicated images; signs of a paper mill; original data or images not available; unreliable results or conclusions.

**Figure 1:** *FOXD2-AS1* is upregulated in cervical cancer tissues and cell lines. **(A)** RT-qPCR was carried out to analyze *FOXD2-AS1* expression in 63 pairs of cervical cancer tissue samples and adjacent noncancerous tissues. *P < 0.05 vs noncancerous tissues. **(B)** The Kaplan–Meier survival curve of patients with cervical cancer classified as low- and high-*FOXD2-AS1* groups based on a median expression level of *FOXD2-AS1*. P = 0.019. **(C)** Expression of *FOXD2-AS1* in four cervical cancer cell lines (HeLa, C-33A, SiHa, and CaSki) and a normal human cervix epithelial cell line (Ect1/E6E7) was determined by RT-qPCR. *P < 0.05 vs Ect1/E6E7 cells.

**Table 1:** Clinical parameters associated with lncRNA *FOXD2-AS1* expression among patients with cervical cancer.

Parameters	*FOXD2-AS1* expression		P value
	High (n = 32)	Low (n = 31)	
**Age**			0.613
<55 years	15	12	
≥55 years	17	19	
**Tumor size**			0.609
<4 cm	21	18	
≥4 cm	11	13	
**Histological grade**			0.305
Well-differentiated tumor tissue	10	14	
Moderately or poorly differentiated tumor tissue	22	17	
**FIGO stage**			0.045
I-II	11	19	
III-IV	21	12	
**Lymph node metastasis**			0.023
No	13	22	
Yes	19	9	
**Depth of cervical invasion**			0.036
<2/3	16	24	
≥2/3	16	7	

The article "Long Noncoding RNA FOXD2-AS1 Promotes the Malignancy of Cervical Cancer by Sponging MicroRNA-760 and Upregulating Hepatoma-Derived Growth Factor" was retracted in 2023. Reasons: duplicated images; signs of a paper mill; original data or images not available; unreliable results or conclusions.

### Inhibition of *FOXD2-AS1* Expression Suppresses Cervical Cancer Cell Proliferation, Migration, and Invasion and Promotes Apoptosis

To reveal the exact roles of *FOXD2-AS1* in the progression of cervical cancer, HeLa and SiHa cell lines, which showed relatively high *FOXD2-AS1* expression among the four cervical cancer cell lines, were selected for functional analysis and were transfected with si-FOXD2-AS1. In the two cell lines, the successful downregulation of *FOXD2-AS1* was confirmed *via* RT-qPCR (**Figure 2A**, P < 0.05). The effect of the *FOXD2-AS1* knockdown on the proliferation of cervical cancer cells was tested by the MTT assay. The data revealed that the knockdown of *FOXD2-AS1* decreased the proliferation of HeLa and SiHa cells (**Figure 2B**, P < 0.05). In addition, during quantitation of apoptotic cells by flow cytometry, si-FOXD2-AS1-transfected HeLa and SiHa cells were found to have a higher apoptosis rate compared with the cells transfected with si-NC (**Figure 2C**, P < 0.05). Furthermore, the cell motility was determined by migration and invasion assays, and the results showed that the migration (**Figure 2D**, P < 0.05) and invasiveness (**Figure 2E**, P < 0.05) of HeLa and SiHa cells obviously decreased after si-FOXD2-AS1 transfection. These observations revealed oncogenic roles of *FOXD2-AS1* in the proliferation, apoptosis, migration, and invasiveness of cervical cancer cells.

**Figure 2:** Knockdown of *FOXD2-AS1* inhibits cervical cancer cell proliferation, migration, and invasion *in vivo* but promotes the apoptosis of these cells. **(A)** *FOXD2-AS1* expression in HeLa and SiHa cells transfected with si-FOXD2-AS1 or si-NC was examined using RT-qPCR. *P < 0.05 vs group “si-NC.” **(B)** The MTT assay was performed for determining the proliferative abilities of HeLa and SiHa cells after transfection with si-FOXD2-AS1 or si-NC. *P < 0.05 vs group si-NC. **(C)** The percentage of apoptotic *FOXD2-AS1*-deficient HeLa and SiHa cells was assessed by flow cytometry. *P < 0.05 vs the si-NC group. **(D, E)** Migration and invasion assays were conducted to analyze the effects of *FOXD2-AS1* inhibition on the migratory and invasive abilities of HeLa and SiHa cells. *P < 0.05 vs group si-NC.

### *FOXD2-AS1* Sponges miR-760 in Cervical Cancer

The mechanisms behind the oncogenic activity of *FOXD2-AS1* in cervical cancer were investigated next. Competitive endogenous RNA is a well-known regulatory role of lncRNA. LncRNAs may sponge certain miRNAs to inhibit the expression of these miRNAs. A bioinformatics tool, namely starBase 3.0, was used to search for the miRNAs that could interact with *FOXD2-AS1* based on the complementarity of bases. MiR-760 (**Figure 3A**) was found to contain a sequence complementary to *FOXD2-AS1*, and this miRNA was selected for verification because miR-760 exerts tumor-suppressive actions in a variety of human cancers (Hu et al., 2016; Liao et al., 2016; Cao et al., 2018; Yan et al., 2018). The luciferase reporter assay was conducted to test this prediction, and the results showed that upregulation of miR-760 (**Figure 3B**, P < 0.05) caused by miR-760 mimic transfection resulted in obvious suppression of the luciferase activity of FOXD2-AS1-WT (P < 0.05); however, the luciferase activity of FOXD2-AS1-MUT stayed unaltered in HeLa and SiHa cells after miR-760 overexpression (**Figure 3C**).

The article "Long Noncoding RNA FOXD2-AS1 Promotes the Malignancy of Cervical Cancer by Sponging MicroRNA-760 and Upregulating Hepatoma-Derived Growth Factor" was retracted in 2023. Reasons: duplicated images; signs of a paper mill; original data or images not available; unreliable results or conclusions.

**Figure 3:** *FOXD2-AS1* serves as a molecular sponge for miR-760 in cervical cancer. **(A)** miR-760 and its predicted binding site in *FOXD2-AS1*. **(B)** RT-qPCR was carried out to determine the transfection efficiency of the miR-760 mimic in HeLa and SiHa cells. *P < 0.05 vs the miR-NC group. **(C)** Relative luciferase activity analyses in HeLa and SiHa cells cotransfected with either FOXD2-AS1-WT or FOXD2-AS1-MUT and either the miR-760 mimic or miR-NC. *P < 0.05 vs the miR-NC group. **(D)** The RIP assay indicated that both *FOXD2-AS1* and miR-760 were immunoprecipitated by the anti-AGO2 antibody. *P < 0.05 vs the IgG group. **(E)** The expression of miR-760 was measured by RT-qPCR in HeLa and SiHa cells transfected with either si-FOXD2-AS1 or si-NC. *P < 0.05 vs the si-NC group. **(F)** RT-qPCR was carried out to quantify the miR-760 expression in 63 pairs of cervical cancer tissue samples and adjacent noncancerous tissue samples. *P < 0.05 vs noncancerous tissues. **(G)** The expression correlation between levels of *FOXD2-AS1* and miR-760 was analyzed in cervical cancer tissues by Spearman’s correlation analysis. R^2^ = 0.4092, P < 0.0001.

The RIP assay indicated that both *FOXD2-AS1* and miR-760 were immunoprecipitated by the anti-AGO2 antibody in HeLa and SiHa cell lysates, suggesting that miR-760 is a *FOXD2-AS1* target (**Figure 3D**, P < 0.05). Next, the expression of miR-760 in *FOXD2-AS1*–deficient HeLa and SiHa cells was determined by RT-qPCR. The downregulation of *FOXD2-AS1* in HeLa and SiHa cells caused significant upregulation of miR-760 expression (**Figure 3E**, P < 0.05). Furthermore, miR-760 expression was notably lower in cervical cancer tissue samples than in noncancerous tissue samples (**Figure 3F**, P < 0.05). Notably, cervical cancer tissue samples manifested an inverse correlation between the expression levels of *FOXD2-AS1* and miR-760 (**Figure 3G**, R^2^ = 0.4092; P < 0.0001). To sum up, *FOXD2-AS1* sponged miR-760 in cervical cancer cells.

The article "Long Noncoding RNA FOXD2-AS1 Promotes the Malignancy of Cervical Cancer by Sponging MicroRNA-760 and Upregulating Hepatoma-Derived Growth Factor" was retracted in 2023. Reasons: duplicated images; signs of a paper mill; original data or images not available; unreliable results or conclusions.

### MiR-760 Functions as a Tumor-Suppressive miRNA in Cervical Cancer Cells

Next, we examined the involvement of miR-760 in the malignant characteristics of cervical cancer. Because miR-760 expression was low in cervical cancer, gain-of-function experiments were performed on HeLa and SiHa cells after miR-760 mimic or miR-NC transfection. The MTT assay and flow cytometry revealed that the ectopic miR-760 expression restricted the proliferation (**Figure 4A**, P < 0.05) and induced apoptosis (**Figure 4B**, P < 0.05) of HeLa and SiHa cells. After that, the migration and invasiveness of HeLa and SiHa cells were tested in migration and invasion assays after overexpression of miR-760. When HeLa and SiHa cells were transfected with the miR-760 mimic, their migratory (**Figure 4C**, P < 0.05) and invasive (**Figure 4D**, P < 0.05) abilities significantly decreased as compared with those of miR-NC–transfected cells. Collectively, these results revealed the tumor-suppressive functions of miR-760 in cervical cancer cells.

**Figure 4:** miR-760 exerts an inhibitory effect on the growth and metastasis of cervical cancer cells *in vitro*. **(A, B)** The proliferation and apoptosis of miR-760 mimic–transfected or miR-NC–transfected HeLa and SiHa cells was evaluated by the MTT assay and flow-cytometric analysis. *P < 0.05 vs the miR-NC group. **(C, D)** Migration and invasion assays were conducted to determine the migratory and invasive abilities of HeLa and SiHa cells overexpressing miR-760. *P < 0.05 vs the miR-NC group.

### HDGF mRNA Is the Direct Target of miR-760 in Cervical Cancer

To elucidate the mechanisms underlying the roles of miR-760 in cervical cancer, bioinformatics analysis was carried out and predicted that the 3′-UTR of *HDGF* mRNA harbors a potential miR-760–binding site (**Figure 5A**). After that, the luciferase reporter assay was applied to determine whether miR-760 can directly target the 3′-UTR of *HDGF* mRNA in cervical cancer cells. As presented in **Figure 5B**, upregulation of miR-760 significantly decreased the luciferase activities of the luciferase plasmid harboring the wild-type 3′-UTR of *HDGF* (P < 0.05) in HeLa and SiHa cells; however, this effect was abrogated when the binding site in the 3′-UTR of *HDGF* was mutated.

**Figure 5:** *HDGF* mRNA is a direct target of miR-760 in cervical cancer cells. **(A)** The wild-type (WT) and mutant (MUT) binding sites for miR-760 in the 3′-UTR of *HDGF* mRNA as predicted by bioinformatics analysis. **(B)** The luciferase reporter assay was performed on HeLa and SiHa cells that were cotransfected with either the miR-760 mimic or miR-NC and a luciferase reporter plasmid carrying the WT or Mut 3′-UTR of *HDGF*. *P < 0.05 vs group miR-NC. **(C)** *HDGF* mRNA expression was assessed by RT-qPCR in 63 pairs of cervical cancer tissue samples and samples of adjacent noncancerous tissues. *P < 0.05 vs noncancerous tissue samples. **(D)** Spearman’s correlation analysis was applied to investigate the relation between miR-760 and *HDGF* mRNA levels in cervical cancer tissue samples. R^2^ = 0.3554; P < 0.0001. **(E, F)** The mRNA and protein levels of HDGF in HeLa and SiHa cells transfected with either the miR-760 mimic or miR-NC were measured by RT-qPCR and western blotting, respectively. *P < 0.05 vs the miR-NC group.

The article "Long Noncoding RNA FOXD2-AS1 Promotes the Malignancy of Cervical Cancer by Sponging MicroRNA-760 and Upregulating Hepatoma-Derived Growth Factor" was retracted in 2023. Reasons: duplicated images; signs of a paper mill; original data or images not available; unreliable results or conclusions.

The relation between miR-760 and HDGF was further examined by quantification of the HDGF expression in cervical cancer tissues. The mRNA level of HDGF was found to be much higher in cervical cancer tissue samples than in noncancerous tissue samples (**Figure 5C**, P < 0.05). HDGF expression was then compared with miR-760 expression in the same cervical cancer tissue samples. A significant inverse correlation was uncovered by Spearman’s correlation analysis (**Figure 5D**; R^2^ = 0.3554; P < 0.0001). Furthermore, RT-qPCR and western blotting revealed that the expression levels of *HDGF* mRNA (**Figure 5E**, P < 0.05) and protein (**Figure 5F**, P < 0.05) were noticeably lower in HeLa and SiHa cells after miR-760 overexpression. Collectively, these results strongly indicated that *HDGF* mRNA is a direct target of miR-760 in cervical cancer cells.

### HDGF Restoration Counteracts the Effects of miR-760 Overexpression on the Malignant Characteristics of Cervical Cancer Cells

MiR-760 was found to act as a tumor-suppressive miRNA in cervical cancer, and *HDGF* mRNA was validated as a direct target of miR-760; hence, the tumor-suppressive actions of miR-760 in cervical cancer cells were next postulated to be mediated by HDGF downregulation. To test this hypothesis, HDGF overexpression plasmid pcDNA3.1-HDGF (pc-HDGF) or the empty pcDNA3.1 plasmid was cotransfected with the miR-760 mimic into HeLa and SiHa cells. Cotransfection with pc-HDGF efficiently reversed HDGF downregulation by the miR-760 mimic in HeLa and SiHa cells, as indicated by western blotting (**Figure 6A**, P < 0.05). After that, we discovered that restoration of HDGF expression obviously attenuated the influence of miR-760 overexpression on the proliferation (**Figure 6B**, P < 0.05), apoptosis (**Figure 6C**, P < 0.05), migration (**Figure 6D**, P < 0.05), and invasiveness (**Figure 6E**, P < 0.05) of HeLa and SiHa cells. In summary, these results supported the hypothesis that miR-760 overexpression restrained the malignant phenotype of cervical cancer cells, at least partly, by decreasing HDGF expression.

The article "Long Noncoding RNA FOXD2-AS1 Promotes the Malignancy of Cervical Cancer by Sponging MicroRNA-760 and Upregulating Hepatoma-Derived Growth Factor" was retracted in 2023. Reasons: duplicated images; signs of a paper mill; original data or images not available; unreliable results or conclusions.

**Figure 6:** HDGF downregulation mediates the effect of miR-760 in cervical cancer cells. The miR-760 mimic was cotransfected with pcDNA3.1-HDGF (pc-HDGF) or the empty pcDNA3.1 plasmid into HeLa and SiHa cells. The transfected cells were harvested and subjected to the following assays. **(A)** HDGF protein expression was confirmed in the indicated cells by western blot analysis. *P < 0.05 vs group miR-NC. ^#^P < 0.05 vs group miR-760 mimic+pcDNA3.1. **(B–E)** Measurement of proliferation, apoptosis, migration, and invasiveness of the above-mentioned cells was performed by the MTT assay, flow cytometry, and migration and invasion assays, respectively. *P < 0.05 vs the miR-NC group. ^#^P < 0.05 vs the miR-760 mimic+pcDNA3.1 group.

### MiR-760 Downregulation Reverses the Effects of *FOXD2-AS1* Silencing on Cervical Cancer Cells

To further test the involvement of miR-760 in the role induced by *FOXD2-AS1* on the oncogenicity of cervical cancer cells, miR-760 inhibitor or NC inhibitor was introduced into *FOXD2-AS1*-deficient HeLa and SiHa cells, followed by investigation of the ability of these cells to proliferate, undergo apoptosis, migrate, and invade. The cotransfection of miR-760 inhibitor, which efficiently silenced miR-760 expression (**Figure 7A**, P < 0.05), weakened the *FOXD2-AS1* knockdown-mediated upregulation of miR-760 (**Figure 7B**, P < 0.05) and downregulation of HDGF protein (**Figure 7C**, P < 0.05) in HeLa and SiHa cells. The effects of *FOXD2-AS1* downregulation on cellular proliferation (**Figure 7D**, P < 0.05), apoptosis (**Figure 7E**, P < 0.05), migration (**Figure 7F**, P < 0.05), and invasion (**Figure 7G**, P < 0.05) were notably attenuated in HeLa and SiHa cells by miR-760 inhibitor cotransfection. These results indicated that *FOXD2-AS1* silencing exerted an inhibitory action on cervical cancer malignancy by targeting the miR-760–HDGF axis.

**Figure 7:** miR-760 knockdown attenuates the biological effects of *FOXD2-AS1* silencing in cervical cancer cells. **(A)** Either the miR-760 inhibitor or NC inhibitor was transfected into HeLa and SiHa cells. At 48 h after transfection, RT-qPCR was carried out to determine transfection efficiency. *P < 0.05 vs the NC inhibitor group. **(B, C)** Si-FOXD2-AS1 along with either the miR-760 inhibitor or NC inhibitor was introduced into HeLa and SiHa cells. The transfected cells were collected and subjected to the determination of miR-760 and HDGF protein levels by RT-qPCR and western blotting, respectively. *P < 0.05 vs the si-NC group. ^#^P < 0.05 vs the si-FOXD2-AS1+NC inhibitor group. **(D–G)** Cellular proliferation, apoptosis, migration, and invasion were investigated by MTT, flow-cytometric, and migration and invasion assays, respectively, in HeLa and SiHa cells cotransfected with si-FOXD2-AS1 and either the miR-760 inhibitor or NC inhibitor. *P < 0.05 vs group si-NC. ^#^P < 0.05 vs group “si-FOXD2-AS1+NC inhibitor.”.

The article "Long Noncoding RNA FOXD2-AS1 Promotes the Malignancy of Cervical Cancer by Sponging MicroRNA-760 and Upregulating Hepatoma-Derived Growth Factor" was retracted in 2023. Reasons: duplicated images; signs of a paper mill; original data or images not available; unreliable results or conclusions.

### Depletion of *FOXD2-AS1* Decreases Cervical Cancer Tumor Growth *In Vivo*

To characterize the influence of *FOXD2-AS1* on tumor growth *in vivo*, an *in vivo* tumorigenicity assay was performed *via* injection of si-FOXD2-AS1 or si-NC-transfected HeLa cells into the flank of nude mice. Si-FOXD2-AS1 HeLa cell–injected nude mice showed slower tumor growth (**Figures 8A**, **B**; P < 0.05) and smaller tumor weight (**Figure 8C**, P < 0.05) than the si-NC HeLa cell-injected ones. In addition, the tumor xenografts of the si-FOXD2-AS1 group featured downregulation of *FOXD2-AS1* (**Figure 8D**, P < 0.05), higher miR-760 expression (**Figure 8E**, P < 0.05), and lower HDGF mRNA (**Figure 8F**, P < 0.05) and protein expression (**Figure 8G**, P < 0.05) relative to those in the si-NC group. Consistently with the *in vitro* findings, downregulation of *FOXD2-AS1* decreased the expression of HDGF *via* reduced sponging of miR-760, thereby inhibiting tumor growth *in vivo*.

**Figure 8:** The *FOXD2-AS1* knockdown inhibits cervical cancer growth *in vivo*. **(A)** A representative image of tumor xenografts from groups “si-FOXD2-AS1” and “si-NC.” **(B)** *FOXD2-AS1*-deficient HeLa cells were injected into nude mice. Then tumor volumes were measured every 2 days starting at 2 weeks after the injection. *P < 0.05 vs group si-NC. **(C)** All nude mice were euthanized at the end of the experiment. The tumor xenografts were resected and weighed. *P < 0.05 vs the si-NC group. **(D–G)** *FOXD2-AS1*, miR-760, *HDGF* mRNA, and HDGF protein levels were quantified in the tumor xenografts derived from si-FOXD2-AS1–transfected or si-NC–transfected HeLa cells.

## Discussion

LncRNAs are a large subgroup of noncoding RNAs that have emerged as regulators of crucial processes in various human cancers including cervical cancer (Aalijahan and Ghorbian, 2019). In recent decades, multiple lncRNAs have been reported to be aberrantly expressed in cervical cancer, and their aberrant expression plays important roles in the aggressive phenotype of cervical cancer (Cui et al., 2017; Dong et al., 2017; Wang et al., 2017). Hence, exploration of the detailed involvement of lncRNAs in cervical cancer and their mechanisms of action is necessary to discover promising targets for the diagnosis and treatment of patients with this cancer. In this study, we for the first time measured *FOXD2-AS1* expression in cervical cancer and determined its clinical value in patients with cervical cancer. Notably, the biological roles and regulatory mechanism of action of *FOXD2-AS1* in cervical cancer were investigated in detail.

The article "Long Noncoding RNA FOXD2-AS1 Promotes the Malignancy of Cervical Cancer by Sponging MicroRNA-760 and Upregulating Hepatoma-Derived Growth Factor" was retracted in 2023. Reasons: duplicated images; signs of a paper mill; original data or images not available; unreliable results or conclusions.

*FOXD2-AS1* is overexpressed in bladder cancer, and upregulation of *FOXD2-AS1* shows a significant correlation with tumor stage and tumor recurrence (Su et al., 2018). The overall survival and progression-free survival of bladder cancer patients with high *FOXD2-AS1* expression is shorter than that of bladder cancer patients with low *FOXD2-AS1* expression (Su et al., 2018). Overexpressed *FOXD2-AS1* is observed in multiple other types of human cancer, including hepatocellular carcinoma (Chang et al., 2018; Zhao et al., 2018; Xu et al., 2019), glioma (Ni et al., 2019), thyroid cancer (Zhang et al., 2018; Jiang et al., 2019; Liu et al., 2019), cutaneous melanoma (Ren et al., 2019), colorectal cancer (Zhu et al., 2018), esophageal squamous cell carcinoma (Bao et al., 2018), and non–small cell lung cancer (Rong et al., 2017). Nevertheless, *FOXD2-AS1* expression status in cervical cancer has been unknown and warrants investigation. In this study, we found that *FOXD2-AS1* expression is high in both cervical cancer tissues and cell lines. Elevated *FOXD2-AS1* HDGF levels were linked with the FIGO stage, lymph node metastasis, and depth of cervical invasion among patients with cervical cancer. Patients with cervical cancer harboring high *FOXD2-AS1* expression showed worse overall survival than those with low *FOXD2-AS1* expression. These findings suggest that *FOXD2-AS1* is a potential biomarker for the diagnosis and prognosis of cervical cancer.

A knockdown of *FOXD2-AS1* inhibits papillary thyroid cancer cell proliferation, migration, invasion, the cancer stem cell-like phenotype, and anoikis resistance *in vitro*; promotes apoptosis; and hinders tumorigenesis *in vivo* (Zhang et al., 2018; Jiang et al., 2019; Liu et al., 2019). In hepatocellular carcinoma, silencing of *FOXD2-AS1* expression suppresses cell proliferation, colony formation, metastasis, and epithelial–mesenchymal transition; induces cell cycle arrest at the G0–G1 transition; and decreases tumor growth and metastasis *in vivo* (Chang et al., 2018; Zhao et al., 2018; Xu et al., 2019). *FOXD2-AS1* also exerts oncogenic actions on carcinogenesis including progression of bladder cancer (Su et al., 2018), glioma (Ni et al., 2019), cutaneous melanoma (Ren et al., 2019), colorectal cancer (Zhu et al., 2018), esophageal squamous cell carcinoma (Bao et al., 2018), and non–small cell lung cancer (Rong et al., 2017). Nevertheless, no studies have focused on specific functional roles of *FOXD2-AS1* in the malignant characteristics of cervical cancer. Herein, we demonstrated that *FOXD2-AS1* knockdown attenuates cervical cancer cell proliferation, migration, and invasion *in vitro*; increased apoptosis; and hindered tumor growth *in vivo*. These observations suggest that *FOXD2-AS1* may be considered an effective target for cervical cancer therapies in the future.

The article "Long Noncoding RNA FOXD2-AS1 Promotes the Malignancy of Cervical Cancer by Sponging MicroRNA-760 and Upregulating Hepatoma-Derived Growth Factor" was retracted in 2023. Reasons: duplicated images; signs of a paper mill; original data or images not available; unreliable results or conclusions.

Exploration of the molecular mechanisms underlying the oncogenic activity of *FOXD2-AS1* is essential for the identification of novel therapeutic methods for patients with cervical cancer. Our investigation of the mechanism revealed that *FOXD2-AS1* may serve as a competitive endogenous RNA for miR-760. This miRNA is overexpressed in ovarian cancer (Liao et al., 2016) and functions as an oncogenic miRNA during cancer progression. On the contrary, miR-760 is underexpressed in hepatocellular carcinoma, non–small cell lung cancer (Yan et al., 2018), colorectal cancer (Cao et al., 2018), and breast cancer (Hu et al., 2016). Functionally, miR-760 is reported to play a tumor-suppressive part in the aggressiveness of these human cancer types. The expression and participation of miR-760 in cervical cancer have been unclear. Our results revealed that miR-760 expression is low in cervical cancer. By contrast, miR-760 overexpression inhibited the malignancy of cervical cancer by suppressing cell proliferation, migration, and invasion and by increasing apoptosis. Therefore, our study for the first time revealed the crucial functions of the *FOXD2-AS1*–miR-760 pathway in cervical cancer.

After that, we explored the mechanisms behind the activities of miR-760 in cervical cancer. Our results identified *HDGF* as a direct target gene of miR-760 in cervical cancer, and downregulation of HDGF turned out to be essential for the biological functions of miR-760 in cervical cancer. HDGF is overexpressed in cervical cancer tissues in comparison with nontumor tissues. Upregulation of HDGF is closely related to lymph-vascular space invasion, lymph node metastasis, recurrence, and advanced grade among patients with cervical cancer (Tsai et al., 2014). HDGF participates in the progression of cervical cancer by promoting cell proliferation, migration, and invasion (Song et al., 2017). The results of the present study revealed that HDGF is directly regulated by the *FOXD2-AS1*–miR-760 pathway in cervical cancer and is involved in multiple cancer-related pathological processes.

The study had two limitations. First, Northern Blot assay was not applied to detect miR-760 expression in cervical cancer. Second, the impact of *FOXD2-AS1* on the occurrence of cervical cancer was not explored in detail. We will resolve the limitations in the near further.

The article "Long Noncoding RNA FOXD2-AS1 Promotes the Malignancy of Cervical Cancer by Sponging MicroRNA-760 and Upregulating Hepatoma-Derived Growth Factor" was retracted in 2023. Reasons: duplicated images; signs of a paper mill; original data or images not available; unreliable results or conclusions.

In summary, the present study shows that *FOXD2-AS1* expression is high in cervical cancer, and this overexpression is associated with poor prognosis. Downregulation of *FOXD2-AS1* inhibits the malignant characteristics of cervical cancer cells by decreasing competitive sponging of miR-760, thereby decreasing HDGF expression. The *FOXD2-AS1*–miR-760–HDGF pathway represents an effective target for the treatment of patients with cervical cancer.

## Data Availability Statement

The datasets used and/or analyzed during the present study are available from the corresponding authors on reasonable request.

## Ethics Statement

The studies involving human participants were reviewed and approved by the ethics committee of The First Affiliated Hospital of Zhejiang Chinese Medical University. The patients/participants provided their written informed consent to participate in this study. The animal study was reviewed and approved by the Institutional Animal Care and Use Committee of The First Affiliated Hospital of Zhejiang Chinese Medical University.

## Author Contributions

XD, QZ, MW, JX, YZ, SZ, and XX have made a significant contribution to the findings and methods. They have read and approved the final draft.

## Funding

Financial support was provided by the Zhejiang Medical and Health Science Technology Project (2015KYA168).

## Conflict of Interests

The authors declare that the research was conducted in the absence of any commercial or financial relationships that could be construed as a potential conflict of interest.
